The article "Determination of Bridge Prestress Loss under Fatigue Load Based on PSO-BP Neural Network" was retracted in 2023. Reasons: unreliable results or conclusions; concerns about the data; concerns about the peer review; concerns about the citations.

# Determination of Bridge Prestress Loss under Fatigue Load Based on PSO-BP Neural Network

**DOI:** 10.1155/2021/4520571

**Published:** 2021-07-12

**Authors:** Yongguang Wang

**Affiliations:** ^1^School of Transportation, Wuhan University of Technology, Wuhan 430063, China; ^2^Zhonggongchengke (Jilin) Engineering Testing Co., Ltd, Changchun 130117, China

## Abstract

During the service period of a prestressed concrete bridge, as the number of cyclic loads increases, cumulative fatigue damage and prestress loss will occur inside the structure, which will affect the safety, durability, and service life of the structure. Based on this, this paper studies the loss of bridge prestress under fatigue load. First, the relationship between the prestress loss of the prestressed tendons and the residual deflection of the test beam is analyzed. Based on the test results and the main influencing factors of fatigue and creep, a concrete fatigue and creep calculation model is proposed; then, based on the static cracking check calculation method and POS-BP neural network algorithm, a prestressed concrete beam fatigue cracking check model under repeated loads is proposed. Finally, the mechanical performance of the prestressed concrete beam after fatigue loading is analyzed, and the influence of the fatigue load on the bearing capacity of the prestressed concrete beam is explored. The results show that the bridge prestress loss characterization model based on the POS-BP neural network algorithm has the advantages of high calculation efficiency and strong applicability.

## 1. Introduction

At present, although some progress has been made in the research of bridge prestress, most construction enterprises have some problems in the process of loss and analysis of bridge prestress under fatigue load. With the development of intelligent technology, the research on the mechanical and bearing capacity of building bridges has also been developed rapidly. In addition, in the modeling and analysis of the bearing capacity of bridge buildings, the advantages of the prestressed design of bridges under fatigue load based on cloud computing technology and intelligent algorithm are more obvious. The development of these technologies also provides opportunities for the research on the combination of the prestressed design and ultimate load performance of the bridge under the action of building stability and fatigue load [1]. Therefore, the mechanical performance analysis and bearing capacity design of the bridge prestressed under fatigue load have become an important index to judge the advanced level of bridge construction field, and there have been studies on the application of neural network algorithms to the determination of prestress loss [2]. On the other hand, how to combine intelligent algorithm and bearing capacity technology to establish a modern and efficient measurement system of prestress loss under fatigue load has become an important development direction [3]. Up to now, a lot of data have been produced in the comprehensive performance analysis and bearing capacity test of the bridge prestress under fatigue load [4]. How to extract, collect, and store the mechanical properties of the bridge through these redundant data has become the main research direction of the research on the mechanical property change and ultimate load effect of the bridge prestress under the fatigue load [5]. Scholars conducted fatigue and postfatigue static load tests on 11 partially prestressed concrete test beams. The results showed that the load-bearing capacity of prestressed concrete beams after fatigue is related to the degree of fatigue damage of the beam body. The ultimate load-bearing capacity of the test beam is basically not affected, while the moderate and severe fatigue damage reduce the ultimate strength of the test beam by 15.2% and 18.0%, respectively [6]. On the basis of model tests, modern researchers analyzed the bearing capacity of bonded and unbonded prestressed concrete beams after cracking and put forward a rapid evaluation model of the bearing capacity after cracking [7]. Through the design of related experiments, it is proved that the improved algorithm has good mechanical properties and ultimate load effect. Based on the characteristics of limit load theory and fatigue design, some scholars have proposed a hierarchical method for mechanical performance analysis and limit load integration [8]. Based on the fatigue damage accumulation theory, according to the mechanical properties of box girder webs under fatigue load, the criteria of roof cracking and web fatigue failure are given, and the fatigue life evaluation method of prestressed concrete box girder bridge webs is proposed [9]. In order to improve the efficiency of mechanical property analysis of bridge prestress under fatigue load and the stability and safety of mechanical property analysis system in the calculation process, a new mechanical property analysis system based on hyperchaotic mapping is proposed [10]. Scholars have verified the effectiveness of the prestressed analysis model system through practice, which is suitable for data mining and data screening of prestressed mechanical analysis under different types of fatigue load [11]. From the perspective of data information theory and traditional classical mechanical stress analysis, researchers put forward that we should pay attention to the development of customized mechanical analysis and modeling of bridge prestress under different types of fatigue load [12]. Based on the fatigue test results of unbonded prestressed concrete model beams, a nonlinear fatigue damage analysis method considering the stress redistribution of steel and concrete under fatigue load is proposed, and a more practical nonlinear fatigue damage analysis method is obtained [13]. Relevant scholars proposed to strengthen the construction and management of cloud cooperation system and realized the integrated construction combined with the bearing capacity system of the whole bridge [14]. The research finds that the prestressed bridge under fatigue load still follows the traditional architectural design concept in design mode, neglecting the innovation of modernism aesthetics and bearing capacity mode [15]. It is found that in the design process of prestressed bridge structure, the prestress of bridge under fatigue load is mainly used to obtain, store, and transfer different data. The efficiency of high precision control and collaborative design of bridge prestress under fatigue load is very low [16]. In conclusion, it can be seen that in the process of design and ultimate load treatment of the bridge prestress mechanical performance analysis model under the current fatigue load, there are problems with high data redundancy, low calculation efficiency, and poor ultimate load effect [17]. And most of them did not involve intelligent algorithms combined with distributed computing technology and did not apply intelligent solutions to the study of prestress loss of bridges [18]. On the other hand, although a lot of basic research has been done on the design and mechanical performance analysis of the bridge prestress under the fatigue load, the research results on the mechanical performance analysis and bearing capacity design of the bridge under different types of fatigue load are relatively few, and there is no strong robust model for limit load effect analysis [19]. Based on this background, this paper studies the method of determining the loss of prestress and modeling the mechanical properties of the bridge under fatigue load based on PSO-BP neural network algorithm.

The article "Determination of Bridge Prestress Loss under Fatigue Load Based on PSO-BP Neural Network" was retracted in 2023. Reasons: unreliable results or conclusions; concerns about the data; concerns about the peer review; concerns about the citations.

This paper studies the application of bearing capacity and mechanical performance analysis model in the optimization of bridge prestress design under modern fatigue loads and is mainly divided into five sections.  Section 1 introduces the research methods of bridge prestress under the action of modernism fatigue load at home and abroad, as well as the research status of the bridge's ultimate load index and mechanical performance analysis.  Section 2 introduces the application thought of POS-BP neural network algorithm in the analysis model of bridge prestress under fatigue load.  Section 3 is based on the commonly used POS-BP neural network algorithm, constructs the mechanical performance analysis model of the bridge prestress under fatigue load based on the POS-BP neural network algorithm, and combines the Gaussian random matrix and the characteristic judgment matrix. The control strategy of the objective function constructs an evaluation index system for the influence of the mechanical properties of the bridge prestress under fatigue load.  Section 4 tests the mechanical performance and ultimate load effect of the bridge prestress under the fatigue load constructed in this paper and evaluates the mechanical analysis and ultimate load effect of the bridge prestress under different types of fatigue loads.  Section 5 draws conclusions and analyzes the shortcomings.

## 2. Application of PSO-BP Neural Network Algorithm in Bridge Prestress Analysis Model under Fatigue Load

PSO-BP neural network algorithm is a multilayer feedforward network trained by error backpropagation algorithm, which is one of the most widely used neural network models. PSO-BP neural network algorithm is different from the conventional algorithm, which is a better multiresource control and calculation strategy [20]. At present, PSO-BP neural network algorithm has been applied in traditional industrial production, control engineering, Internet of things system control, traffic data analysis, image processing and precise control of national defense space equipment, scheduling and traveling salesman problem, semantics, chemical phase equilibrium, clustering, dynamic problem, rigid image registration problem, parameter selection, and material mechanical property analysis. It has been widely used in protein folding and other fields [21]. Generally speaking, although PSO-BP neural network algorithm has many layers of meaning, its basic meaning of optimization inspiration is consistent, that is, the algorithm has strong expansibility and need and can provide a new idea for optimization analysis of complex problems in different industries [22]. The conventional mathematical calculation idea of PSO-BP neural network algorithm is shown in Figure 1. The core of PSO-BP neural network algorithm is that it can coordinate many local resources of different dimensions. At the same time, it is also an innovation in the field of local optimization algorithm after Internet and computer. Heuristic optimization algorithm is a major innovation in the information age [23].

At present, the PSO-BP neural network algorithm is widely used in the optimization analysis of the mechanical properties of materials. In the mechanical property analysis system for different types of bridge buildings, most of them are based on the PSO-BP neural network algorithm for approximate simulation solution [24]. The objective problem optimization strategy of PSO-BP neural network algorithm is to provide effective approximate solution algorithm and optimal calculation strategy for high-dimensional problems with large amount of data and improve the optimization efficiency of overall mechanical performance analysis and utilization of storage resources. The commonly used characteristic analysis factors are shown in Table 1.

The article "Determination of Bridge Prestress Loss under Fatigue Load Based on PSO-BP Neural Network" was retracted in 2023. Reasons: unreliable results or conclusions; concerns about the data; concerns about the peer review; concerns about the citations.

## 3. Study on Determination of Prestress Loss of Bridge under Fatigue Load

### 3.1. Analysis Model of Bridge Prestressed Ultimate Load Performance Based on PSO-BP Neural Network Algorithm

The traditional analysis method of bridge prestress performance is based on the classical Newton mechanics principle, which cannot carry out the visual overall simulation analysis of its stress process [25]. Therefore, in the process of analyzing the ultimate load performance of bridge prestress under fatigue load, we select four characteristic parameters related to the efficiency of mechanical performance analysis and design an efficient and intelligent adaptive analysis model for ultimate load performance of bridge construction. The judgment factor expression *f*(*x*) in this process is as follows:

(1) $$\begin{array}{c} f\left(x\right)=\frac{\sqrt{x+3}}{x^{3}+2x^{2}+5x-1}, \end{array}$$

where *x* is the prestress load, and *h*(*x*) is the expression of neural node factor:

(2) $$\begin{array}{c} h\left(x\right)=\frac{x^{3}+x+3}{x^{3}+6x^{2}+8x+3}. \end{array}$$

The adaptive analysis model can realize the unified management of the basic parameter information source of bridge prestress under different types of fatigue load, the local difference analysis of bridge prestressed mechanical properties under fatigue load is realized, and the coupling coefficient *η* is as follows:

(3) $$\begin{array}{c} \eta =\sqrt{\frac{x^{3}+x^{2}+2}{x^{4}+7x^{3}+8x^{2}+10x}}. \end{array}$$

Then, the PSO-BP neural network algorithm is used for intelligent control and feedback correction, so as to realize the analysis of bridge prestressed mechanical properties and data storage under different types of fatigue load. After completing the above basic mechanical performance analysis, according to the collection process of ultimate load performance analysis data of bridge prestress under different types of fatigue load, the vector differences in the eigenvalues of different data, and the structural characteristics of the data, the matrix difference and other different characteristic description values are analyzed; the corresponding characterization function *w*(*x*) is as follows:

(4) $$\begin{array}{c} w\left(x\right)=\frac{\sqrt{x^{3}+x^{2}+2/x^{4}+7x^{3}+8x^{2}+10x}}{x^{2}+3x}. \end{array}$$

Then, the intelligent optimization process and deep mining process based on PSO-BP neural network algorithm are used to realize the mechanical and ultimate load performance analysis and law analysis of bridge prestress under fatigue load in different types and different structural design methods. The finite element simulation analysis process of bridge prestress under fatigue load is shown in Figure 2.

The article "Determination of Bridge Prestress Loss under Fatigue Load Based on PSO-BP Neural Network" was retracted in 2023. Reasons: unreliable results or conclusions; concerns about the data; concerns about the peer review; concerns about the citations.

PSO-BP neural network algorithm is used to analyze the mechanical properties of bridge prestress under different fatigue loads, eliminate redundant data, extract effective information, classify data and optimize storage strategy, which is the necessary process of the experiment, and achieve the height classification according to the similarity degree in the design of ultimate load of the bridge prestress under the fatigue load. The data collection, information mining, and feature extraction of different ultimate load performance analysis data are realized. When the mechanical performance analysis data of the bridge prestress under repeated fatigue load are reused or the invalid information is analyzed repeatedly, the feedback control strategy of PSO-BP neural network algorithm will be adopted to control the different types of data information according to the known absorption coefficient requirements. Then, the process of collecting the effective data, feature classification, extracting mechanical information, and quantitative characterization of the bridge prestress under fatigue load is completed. The corresponding data reference range is shown in Table 2.

The operation analysis process of its performance is shown in Figure 3.

### 3.2. Working Process and Calculation Steps of Optimization Analysis of Bridge Prestressed Mechanical Properties and Ultimate Load Effect under Fatigue Load

The PSO-BP neural network algorithm used in this study is a discrete PSO-BP neural network algorithm. The basic steps of the analysis of the mechanical properties of bridge prestress under fatigue load are as follows.

In the first step, in the process of analyzing the mechanical properties of the bridge prestress under the fatigue load of known types and structural shapes, there is often a problem that the error is too large in the process of analyzing the mechanical properties of the bridge prestress under the fatigue load due to the deviation of the discrete neural network algorithm in setting the standard mechanical parameters. Therefore, in the analysis process of the bridge prestress under the fatigue load with known type, structure shape, and thickness information, combined with the classical strategy analysis method based on traditional Newton mechanics, the PSO-BP neural network algorithm is used. Based on the random data eigenvector generated in the bridge prestress database under fatigue load collected by the finite element simulation system, the problem of large mean square error of bridge prestress under different types of fatigue load is solved by hierarchical closed-loop regulation [26]. The judgment factor expression *f*(*x*) in this process is
  (5) $$\begin{array}{c} f\left(x\right)=\frac{\sqrt{x+3}}{x^{3}+2x^{2}+5x-1}. \end{array}$$
In order to solve the problem of low cooperation efficiency in the distributed calculation of PSO-BP neural network algorithm for the collection, processing, and classification of bridge prestress data under fatigue load, this study combines the mechanical performance analysis idea based on neural network algorithm and particle swarm optimization algorithm. By simulating the “multiple PSO neural node operation network” in the process of “neural node transfer” modeling and drawing, the evaluation basis of the mechanical performance analysis efficiency of bridge prestress under fatigue load is constructed, so as to realize the performance analysis and result storage of bridge prestress under different fatigue loads. The simulation analysis results are shown in Figure 4. The simulation results of PSO-BP neural network algorithm are better than those of PSO, BP, and NN.
In the second step, when the mechanical and ultimate load performance analysis model analyzes the corresponding datasets of bridge prestress under different fatigue loads, its ultimate load and prestress data identification rules will attribute the unknown data information to the same data cluster group according to the corresponding mechanical eigenvalues. When the characteristic values of any two data cluster groups in the data of bridge prestressed mechanical performance analysis under different types of fatigue load are different, it means that the characteristic information of the two kinds of data is greatly different. When the mechanical performance analysis model is used to analyze and solve the ultimate load of bridge prestress under different fatigue loads, the selection of eigenvector is limited by the stability, and its modulus length is determined by the modulus length of eigenvector *y*. The corresponding basic strategy function *p*(*x*) is as follows:
  (6) $$\begin{array}{c} p\left(x\right)=\frac{y+\sqrt{f\left(x\right)}}{f\left(x\right)+5x-1}. \end{array}$$
The selected eigenvector *y* needs fitting analysis to know the stability effect of the mechanical property analysis model. Therefore, the equation needs to be optimized and decoupled. The fitting analysis function is
  (7) $$\begin{array}{c} k\left(x\right)=\frac{p\left(x\right)+\sqrt{f\left(x\right)}}{p\left(x\right)+f\left(x\right)+y}. \end{array}$$
In the third step, in the process of mechanical and ultimate load performance analysis of bridge prestress under different fatigue loads, it is necessary to carry out targeted compensation for the placement characteristics of bridge prestress under different types of fatigue loads. The mechanical analysis function *l*(*x*) before compensation is
  (8) $$\begin{array}{c} l\left(x\right)=\sqrt{\frac{k^{2}\left(x\right)+\sqrt{p\left(x\right)}}{k^{2}\left(x\right)+f^{2}\left(x\right)}}. \end{array}$$
The mechanical analysis function *l*′(*x*) after compensation is
  (9) $$\begin{array}{c} l^{\prime }\left(x\right)=1+\sqrt{\frac{k^{2}\left(x\right)+\sqrt{p\left(x\right)}}{k^{2}\left(x\right)+f^{2}\left(x\right)-h\left(x\right)}}. \end{array}$$
When the differential evolution strategy is used to analyze the mechanical properties of different datasets, three common mechanical properties analysis rules will be randomly selected. The three analysis rule functions *e*(*x*), *r*(*x*), and *u*(*x*) are
  (10) $$\begin{array}{c} e\left(x\right)=\frac{\sqrt{l^{2}\left(x\right)+l\left(x\right)-x}}{x},\\ r\left(x\right)=\frac{\sqrt{l^{2}\left(x\right)+2l\left(x\right)-3x}}{2x},\\ u\left(x\right)=\frac{\sqrt{3l^{2}\left(x\right)+4l\left(x\right)-5x}}{6x+1}. \end{array}$$

Among them, different data structures will be obtained under different rules of mechanical properties and ultimate load effect analysis. In order to extract the characteristics of different types of mechanical data and analyze effective data, it is necessary to simulate the prestressed stress of the bridge under these different types of fatigue loads on the mechanical and ultimate load levels [27]. The overall operation process of the finite element simulation analysis system is shown in Figure 5. It can be seen from Figure 5 that under different fatigue loads, the simulation results of bridge dynamic analysis are different, but the laws are the same and show fluctuations in a certain range.

The article "Determination of Bridge Prestress Loss under Fatigue Load Based on PSO-BP Neural Network" was retracted in 2023. Reasons: unreliable results or conclusions; concerns about the data; concerns about the peer review; concerns about the citations.

### 3.3. Innovation Analysis of Bridge Prestress Loss Determination Model Based on PSO-BP Neural Network Algorithm

The innovation of this paper lies in the application of neural network algorithm and bearing capacity design idea to the modeling and analysis of bridge mechanical properties. On this basis, we can make full use of the basic information and characteristic parameters of bridge prestress under different types of fatigue load in Internet database. The unified mechanical performance analysis of bridge prestress under fatigue load is realized. The similarity degree between the comparison columns (the mechanical characteristics of bridge prestress under different types of fatigue load) and the reference columns (the known mechanical characteristics of bridge prestress under standard fatigue load) and the agreement degree of the expected index (the effective data of bearing capacity level) are quantitatively described by the characteristic coefficient. The quantitative index is used to sort the influence degree of the efficiency of the bridge prestressed ultimate load performance analysis model under fatigue load, which can effectively realize the optimal control and ultimate load design of the bridge prestressed under different types of fatigue load through different control methods.

## 4. Result Analysis and Discussion

### 4.1. Experimental Process of Determining and Analyzing Prestress Loss of Bridge under Fatigue Load

In order to study the deflection and flexural stiffness degradation of the prestressed concrete structure under fatigue loading after cracking, FTG-3 and FTG-4 beams were subjected to 2 million constant-amplitude fatigue loading tests and the crack growth at the cracks of the beams was observed. Through the formation of new cracks and the deflection of model beam, the development rules of mid-span deflection, steel strain, and concrete strain, as well as the corresponding crack width and strain amplitude under fatigue load, are studied and analyzed. In the experiment, the experimental objects involved in this study are the samples of the bridge prestressed optimization design under the fatigue load of different types of structures. It can quickly collect, analyze, extract, transform, and store the mechanical and ultimate load performance of the bridge prestressed under fatigue load (the finite element simulation process includes at least 100 information of mechanical change and dynamic limit load effect fitting). By analyzing other characteristics of prestress under different structural fatigue loads, different ultimate load characteristics are obtained. And cloud records are obtained, so as to achieve high-precision performance simulation. Then, based on the analysis of mechanical properties, the ultimate bearing capacity of prestressed bridge under different types of fatigue load is achieved. The experimental data are shown in Table 3.

In this way, in the follow-up process of big data analysis, we can query, call, and determine the ultimate load scheme with high accuracy and high efficiency (the application scenarios of different types of ultimate load schemes correspond to the bridge prestress under the fatigue load of different mechanical properties), so that under the big data collection and storage system, the, To achieve the accurate distribution of bridge prestress design process under each fatigue load, improve the integrity of the ultimate load analysis and prestress loss determination. The preliminary experimental analysis results of the bridge prestress loss determination model under the fatigue load are shown in Figure 6.

The article "Determination of Bridge Prestress Loss under Fatigue Load Based on PSO-BP Neural Network" was retracted in 2023. Reasons: unreliable results or conclusions; concerns about the data; concerns about the peer review; concerns about the citations.

### 4.2. Experimental Results and Analysis

The experimental group is the bridge prestress change and loss under different fatigue loads, and the control group is the bridge prestress of different types of the same structure and the same type of different structures under fatigue loads with known ultimate load effect data. The error of the intelligent optimization design model is analyzed by the experimental process of ultimate load optimization and three groups of known ultimate load performance parameters. The error is shown in Table 4.

The experimental data analysis results of the experimental data are shown in Figure 7.

It can be seen from in Figure 7, that the analysis efficiency and key parameter extraction efficiency of the PSO-BP neural network algorithm under fatigue load are better than those under normal load. Therefore, the algorithm can meet the mechanical performance analysis and ultimate load design of bridge prestress under general fatigue load. In terms of data processing effect of bridge structure reliability, the calculation complexity of the model based on the PSO-BP neural network algorithm for prestress loss analysis and stability performance analysis is low, the effective data acquisition speed is fast, and the state tracking difficulty is low.

## 5. Conclusion

The traditional fatigue load has some problems such as bad ultimate load effect and poor mechanical performance. Based on this, this paper designs the mechanical and ultimate load performance analysis model based on PSO-BP neural network algorithm and studies the process of prestressed design and mechanical performance modeling of bridge under the action of modern fatigue load based on ultimate load. The paper analyzes structural stability, mechanical performance, ultimate load effect, and external aesthetic feeling of the prestressed bridge under the action of conventional fatigue load. The mechanical properties of the prestressed bridge under different fatigue loads are evaluated by using the finite element simulation strategy, and the method can realize adaptive modeling of the mechanical properties and ultimate load effects of the bridge prestress under the fatigue load and realize the diversified analysis and aesthetic design. Finally, the mechanical properties and the application effect of ultimate load of the bridge prestressed under different fatigue loads are analyzed by combining the known characteristics of bridge building and designing the relevant experiments. The experimental results show that the mechanical performance analysis model based on PSO-BP neural network algorithm has the advantages of high calculation efficiency and good mechanical performance simulation effect and can play an effective role in the design of bridge prestress under fatigue load. But this study only considers the loss determination, mechanical properties, and ultimate load effect analysis process of bridge prestress under the action of modern fatigue load and does not consider its reliability factors in other aspects, so deep optimization research can be carried out.

The article "Determination of Bridge Prestress Loss under Fatigue Load Based on PSO-BP Neural Network" was retracted in 2023. Reasons: unreliable results or conclusions; concerns about the data; concerns about the peer review; concerns about the citations.

## Figures and Tables

**Figure 1:** PSO-BP neural network model ideas.

**Figure 2:** The finite element simulation analysis process of the mechanical properties of the bridge prestress.

**Figure 3:** The calculation and analysis process of bridge prestress performance.

**Figure 4:** Performance test of different neural network algorithms at different stages.

**Figure 5:** Calculation results under the finite element simulation analysis system.

**Figure 6:** Preliminary experimental analysis results.

**Figure 7:** Experimental result chart.

**Table 1:** Common indicators and data range.

Common factor indicators	Quantitative indicators
Degree of error	1.5–3.6
Data group	2–17
Neural node	5–9

**Table 2:** Index reference data range.

Common factor indicators	Quantitative indicators
Effective data collection	85%–96%
Feature classification	1–20
Mechanical information extraction	0.25–0.98
Multifactor quantitative characterization	52–100

**Table 3:** Preliminary experimental data results.

Group information	Result
Fatigue load effect 1	0.96
Fatigue load effect 2	0.98
Fatigue load effect 3	0.68

**Table 4:** Error analysis of experimental results.

Group information	Experiment error
Fatigue load effect 1	0.04
Fatigue load effect 2	0.02
Fatigue load effect 3	0.12
From the error reference range	0.01–0.25

## Data Availability

The data used to support the findings of this study are available from the corresponding author upon request.
